This article has been retracted.

# Early Physical Linear Growth of Small-for-Gestational-Age Infants Based on Computer Analysis Method

**DOI:** 10.1155/2021/7227928

**Published:** 2021-10-16

**Authors:** Li Ruixiang, Yin Mingrong, Cui Li, Zheng Rongxiu

**Affiliations:** ^1^College of Clinical Medicine, Tianjin Medical University, Tianjin 300070, China; ^2^Pediatric Department, Affiliated Hospital of Weifang Medical University, Weifang 261031, Shandong, China; ^3^Pediatric Department, Tianjin Medical University General Hospital, Tianjin 300052, China

## Abstract

This article proposes that machine learning can break through the technical limitations of the linear growth test for the early physique of infants smaller than gestational age and can accurately calculate and predict the consequences of the disease. For testing the linear growth of the early physique of infants smaller than gestational age, the data collection and judgment are carried out according to the computer analysis method. Experimental results show that 47.3% of infants younger than gestational age may have suffocation. The experimental subjects designed in this study are small-for-gestational-age infants who were hospitalized in the neonatal intensive care unit from January 2020 to January 2021. According to the relationship between gestational age and birth weight, the survey subjects were divided into two groups: early group and late group. Male and female small-for-gestational-age infants accounted for 68% and 32%, respectively. Among them, the proportion of early gestational age was the most, with more boys than girls, and sick singleton was more than twins. In the early group, the incidence was 52.1% for neonatal asphyxia, 22.5% for feeding intolerance, 14.8% for intracranial hemorrhage, 6.3% for scleredema, 24.7% for neonatal hyperbilirubinemia, 24.6% for hypoglycemia, 1.1% for apnea, and 3.2% for respiratory distress syndrome. Infants develop differently at different stages of corrected gestational age. The incidence of low body weight (6%) after correction for 3 months was significantly reduced compared with correction for gestational age, and the difference was statistically significant (*P* < 0.05). The nutrient absorption of infants younger than gestational age can promote physical catch-up growth, physical development, and neurodevelopment. Therefore, the physical growth of infants younger than gestational age requires supplementation that focuses on nutrition.

## 1. Introduction

Newborn birth weight can reflect the country's social and economic development. With the change in lifestyle, the incidence of small-for-gestational-age infants increases. SGA can bring undesirable consequences, such as short stature, psychosocial problems, and metabolic-related diseases, including hyperlipidemia, type 2 diabetes, and cardiovascular diseases. People are paying more and more attention to the physical health of infants and young children. Once a newborn has a disease and is not treated in time, it will not only lead to an increase in the mortality but also lead to many complications during the perinatal period. At the same time, in tracking the puberty of these newborns, a large part of the babies are far behind other normal newborns of the same age in terms of intelligence, height, weight, and hearing. Vision and many other aspects are obviously lagging behind normal children. Small-for-gestational-age infants, also known as intrauterine growth retardation infants or small sample infants, refer to newborns whose birth weight is lower than the 10th percentile of the average weight of the same gestational age or lower than the two standard deviations of the average weight of the same gestational age. These newborns not only have high risk in perinatal period but also have a series of problems in school age and in adulthood.

There are many results on the physical growth of infants younger than gestational age. For example, Huang et al. assessed the growth trend of full-term small-for-gestational-age babies from birth to 2 years in Chengdu, China. They conducted prospective follow-up of full-term SGA babies from birth to 2 years. They also monitored body weight, length, and head circumference at 3, 6, 12, 18, and 24 months. Catch-up growth and growth rate are measured using standardized scores and Δ*z* scores. There is no significant difference in weight or length at birth between boys and girls [1]. Zhong studies the difference in growth and metabolism between small for gestational age (SGA) and suitable gestational age (AGA). He divided them into SGA group and AGA group according to the correlation between gestational age and birth weight. The general condition, physical development and blood biochemical indexes of the two groups of patients were compared [2]. Zhao et al. aimed to determine whether serum uric acid is a suitable predictor of preeclampsia in women with pregnancy-induced hypertension and in small-for-gestational-age infants. They used uric acid z-score and binary logistic regression analysis to establish the relationship between serum uric acid and the chance of developing pre-eclampsia and having a small-for-gestational-age infant. The results showed that elevated serum uric acid will increase the chance of pregnancy-induced hypertension progressing to pre-eclampsia and subsequent delivery of small-for-gestational-age infants [3]. Specifically, the perinatal mortality of children with SGA is much higher than that of normal weight newborns, and the risk of disease is also increased accordingly. At the same time, these children are also prone to cognitive impairment and learning ability decline when they grow up to school age. After adulthood, the adult lifetime height of many of them will be lower than 2 standard deviations of the normal population.

This article first conducts a simple understanding of infants younger than gestational age, mainly from its definition, problems, etiology, clinical manifestations, treatment methods, classification, prognosis, and so on. Secondly, use computer analysis technology to analyze and predict data for infants smaller than gestational age. Then, they studied the relationship between physical growth and growth rate, collected relevant data, and conducted experimental investigations. Finally, the experimental results are obtained.

## 2. The Linear Growth of the Early Physique of Small-for-Gestational-Age Infants Based on Computer Analysis Method

### 2.1. Small for Gestational Age

#### 2.1.1. Definition

Small-for-gestational-age babies usually indicate that the birth weight of newborns below the 10th percentile of the birth weight of the same gestational age has a high incidence. This part of newborns not only has a very high risk in the perinatal period but also have a series of problems in the school age and adulthood [4, 5].

#### 2.1.2. Problem

1. The mortality rate is higher than that of normal fetuses, and there will be many complications during the perinatal period, including aspiration pneumonia, hypoglycemia, intracranial hemorrhage, asphyxia, hyperbilirubinemia, hypothermia, malnutrition, and the like. It is a more common complication.
2. Small-to-gestational age diseases not only affect the fetal stage but also their growth stage. A large part of the babies are far behind other normal newborns of the same age in terms of body and intelligence after birth. They may have symptoms, such as respiratory infections, diabetes, obesity, short stature, neurocognitive impairment, and poor educational outcomes [6, 7].

#### 2.1.3. Cause

Premature rupture of membranes does not occur in pregnant women with intrauterine infection, and persistent intrauterine infection causes intrauterine growth retardation. Due to the spasm of the small arteries of the umbilical artery, it hinders the blood exchange between the fetus and the mother, causing insufficient blood supply to the fetus, affecting the growth and development of the fetus, resulting in SGA [8, 9].

#### 2.1.4. Clinical Manifestations

1. Malnutrition, weight loss, thinner subcutaneous fat, and dry skin.
2. Hypoglycemia, about one-third of the children will have hypoglycemia within 3 days after birth.
3. Symptoms caused by intrauterine hypoxia, such as amniotic fluid pollution, jaundice, dyspnea, and encephalopathy.
4. Acidosis: metabolic acidosis is caused by tissue hypoxia and hypoxic metabolism.
5. Symptoms of intrauterine infection: hepatosplenomegaly, prolonged jaundice, and retinal choroiditis.
6. Low stress response and low adrenal cortex function.
7. Maternal severe pregnancy complications can affect fetal development. Maternal gestational hypertension (HDCP), multiple pregnancy, and oligohydramnios are the common causes of SGA in late preterm infants. Some pregnant women with intrauterine infection did not have premature rupture of membranes, but persistent intrauterine infection caused intrauterine growth retardation. Systemic arteriolar spasm.

#### 2.1.5. Treatment

In addition to correcting malnutrition and preventing hypoglycemia, growth hormone can accelerate the growth of children with SGA. Growth hormone therapy can significantly increase the height of children with SGA [10, 11]. Some data believe that GH treatment can significantly increase the height of children with SGA and reduce the standard deviation score of height lag. It increases the fastest in the first year of treatment. Its effect positively correlated with the treatment dose, weight, and average height of parents, and negatively correlated with the age of starting treatment. Among them, GH dose has the largest relationship, followed by the age of starting treatment. The growth response in the second year is related to the growth rate in the first year, the age of starting treatment, and GH dose, of which the first one has the greatest relationship.

#### 2.1.6. Prognosis

*(1) Near-Term Prognosis*. Hypoglycemia and metabolic acidosis, polycythemia, meconium aspiration syndrome.

*(2) Long-Term Prognosis*. Physical growth and development. The physical growth and development of full-term infants in terms of height, weight, and head circumference are significantly behind that of normal full-term infants, but there is no difference in bone age and the development of sexual organs [12, 13].

Hypoxic effects of cerebral palsy can affect the generation of DNA in the cells and decrease the number of cells. This effect is most prominent in brain cells, and it is the main reason for the high incidence rate of functional neurological disorders in SGA children, such as language and intellectual impairment and visual and hearing impairment.

#### 2.1.7. Classification

According to the weight index and the ratio of body length to head circumference, SGA is divided into two types: symmetrical type and nonsymmetrical type. The well-proportioned type mostly occurs in the first trimester, and the brain development is damaged to the same degree. The asymmetric type mostly occurs in the third trimester, and the brain development is relatively unaffected, but it is prone to hypoglycemia [14–16].

Nonsymmetrical type: its mass index is less than 2.00 (gestational age is less than or equal to 37 weeks) or less than 2.20 (gestational age is greater than 37 weeks), and the ratio of body length to head circumference is less than 1.36. It is often caused by maternal nutritional factors and vascular diseases, such as pre-eclampsia, chronic gestational hypertension, and uterine abnormalities. Injury occurs in the third trimester of pregnancy. During the period of rapid fetal growth, the decrease of fetal body mass is related to body length. The decrease of head circumference is disproportionate, that is, the body mass is less than the expected gestational age, whereas the body length and head circumference are consistent with the expected gestational age, and the brain development is often not affected.

#### 2.1.8. Comparison

The short-term and long-term prognoses of SGA are quite different from that of AGA. There is high incidence of neonatal asphyxia, neonatal scleredema, neonatal hypoxic ischemic encephalopathy (HIE), congenital malformations, neonatal feeding intolerance, and neonatal hyperbilirubinemia. The incidence of diseases such as intracranial hemorrhage is significantly higher in SGA than that in AGA, and the fatality rate in SGA is much higher than that in AGA.

SGA's organizational ability, sense of direction, and cognitive ability in childhood are lower than those in AGA, and SGA in preadolescence is also trapped in a difficult learning situation. In terms of energy metabolism, SGA may cause diseases such as insulin resistance, obesity, and hyperlipidemia in adulthood. The poor short-term and long-term prognoses of SGA suggest that more attention should be paid to SGA intervention. In late preterm infants, small-for-gestational-age infants have more complicated etiology, more complications, and worse short-term and long-term quality of life [17].

### 2.2. Predicting Infants Small for Gestational Age

In recent years, deep learning has emerged as a part of machine learning. Both in terms of data feature learning and prediction effect, it has shown a higher ability than traditional machine learning. Deep learning avoids these shortcomings of traditional learning. It has the ability to automatically extract features, and at the same time, it can make nonlinear changes to features, which are of great help to the prediction of the model later. Regarding the problem of disease prediction in small-for-gestational-age infants, from the initial prediction of a single physical examination index to the traditional machine learning that integrates multiple examination results to predict the disease, it is impossible to solve the problem of predicting the time-consuming and accurate rate of disease in small-for-gestational-age infants. The problem is not high. After the initial “low-level” feature representation is gradually transformed into “high-level” feature representation through multilayer processing, complex classification and other learning tasks can be completed with “simple model.” Thus, deep learning can be understood as feature learning or representation learning.

In the application of traditional shallow learning algorithms, researchers and developers need to rely on human experience and professional common sense to construct relevant features before putting features into the model. At the same time, the features after model learning are all single-layer features, and nonlinear advanced features cannot be extracted. In addition, a lot of manual screening is required. With the development of science and technology, deep learning has become one of the most effective prediction methods in the field of disease prediction. Deep learning can effectively abstract low-level features into high-level features, avoiding the inaccuracy and time-consuming defects of traditional machine learning that require manual construction of features. Therefore, this article proposed a method based on deep learning to predict small-for-gestational-age infants' diseases. Because this article is based on SGA disease prediction based on deep learning, it is very necessary to understand neural network knowledge. Typical deep learning models include revolutionary neural network, DBN, and stacked auto encoder network models. In addition, DBN can be interpreted as a Bayesian probability generation model, which is composed of multiple layers of random hidden variables. The upper two layers have undirected symmetric connections, the lower layer obtains top-down–directed connections from the upper layer, and the state of the lowest cell is the visible input data vector.

The neuron formula is

(1) $$\begin{array}{c} \text{g}=w\left(\overset{m}{\underset{i=1}{\sum }}\lambda_{i}a_{i}-y\right). \end{array}$$

The feedforward propagation algorithm is to calculate the output value of each neuron using the weights on the connections that have been set and the output formula in the neuron mentioned above as

(2) $$\begin{array}{c} \text{g}=w\left(\overset{m}{\underset{i=0}{\sum }}\lambda_{i}a_{i}\right). \end{array}$$

Autoencoder is an algorithm that allows the model to restore the original data through training. In order to realize the reproduction of the original data, the autoencoder must mine and extract the potential data laws of the original data during the training process.

Recurrent neural networks are mainly used to deal with sequence related problems. The calculation process is as follows:

step 1: *a*(*t*) represents the input at time *t* (*t* = 0,1,2,3, ...);
step 2: *V*_*t*_ is the neuron at time *t* in the hidden layer. The calculation *V*_*t*_ is performed based on the output of the previous network layer and the input of a neuron in the same hidden layer.
  (3) $$\begin{array}{c} V_{t}=w\left(Q*a_{t}+P*V_{t-1}\right). \end{array}$$
step 3: *R*_*t*_ is the output at time *t*. *R*_t_=Soft max(*K∗V*_*t*_). The hidden layer state *V*_*t*_ is the state of the neuron, including the output of the previous hidden layer and the output of a neuron on the same hidden layer. The output *R*_*t*_ of the output layer is only related to the output *v*(*t*). Note that Softmax logistic regression model is a generalization of logistic regression model in multiclassification problems. In multiclassification problems, class label *y* can take more than two values. Softmax regression is supervised, and it will be combined with deep learning and unsupervised learning methods.

Noise reduction autoencoder process (Figure 1):

### 2.3. Physique Linearly Catches up with Growth Rate

Physical examination including height, finger pitch, sitting height, weight, blood pressure, spine, deformity, and intelligence tests should be performed if there is a delay in growth and development. Growth rate is an important indicator to measure whether catch-up growth occurs. At the same time, growth rate is an important content of physical growth assessment, and it can dynamically reflect the physical growth of infants over a period than growth level.

#### 2.3.1. Factors Affecting the Growth Rate of SGA

1. SGA requires higher protein to maintain normal physical growth but does not require higher energy than the recommended value. A relatively low-energy, high-protein diet can ensure that the body mass index (BMI) of SGA remains in an appropriate range. On the premise of ensuring normal physical growth, a suitable low-energy, high-protein diet may be a better choice for SGA.
2. The growth rate of SGA is not only affected by nutritional factors but also regulated by other factors such as heredity and endocrine. Body weight, body length, and head circumference growth rate of 0–3 months old and 3–6 month-old SGA are not related to the average daily energy and daily protein intake. Due to the large energy and protein deficits accumulated in preterm infants, despite the active parenteral and enteral nutrition support in the early postnatal period, the growth curve will still deviate significantly, and SGA in preterm infants is more likely to have adverse growth outcomes. Because it is simultaneously affected by the two factors of premature delivery and SGA, it is more prone to ectopic growth retardation.

#### 2.3.2. Dynamic Changes of SGA Growth Rate within 6 Months of Age

The catch-up growth of SGA can occur in any growth period of infancy, preschool, school age, or adolescence, but most catch-up growth occurs within 2 years of age.

1. Under the premise that energy and protein can ensure normal physical growth requirements, those who accelerate growth to a certain growth level during a certain period may not continue to grow along the growth curve at that level afterwards; although the SGA catches up with growth earlier, after that, there may not necessarily be continuous catch-up growth.
2. The weight and length of SGA in the early postnatal period are not always growing along a specific growth curve but a dynamic process. The reason for this change in growth rate in the early postnatal period of SGA, except for factors such as nutrition and disease, may be that the physical growth of early childhood is strongly affected by genetic factors, and the weight or length tends to return to a level equivalent to genetic factors.

The height in infancy is less correlated with the height in adulthood. Due to the instability of linear growth, the growth level and catch-up growth in the early life of SGA may not be a good predictor of the final height level, so it is necessary to dynamically monitor the physical growth of SGA.

Through research, it is found that the smaller the birth weight of SGA, the faster the weight growth rate at 0–6 months of age; the smaller the birth length of SGA, the faster the growth rate of body length at 0–3 months of age, but the body length at 3–6 months of age growth rate has nothing to do with birth length. The younger the gestational age, the faster the weight and length of SGA at 0–3 months of age will grow, but the growth rate at 3–6 months of age has nothing to do with gestational age. There are also gender differences in physical growth. Male SGA infants with low birth weight have a significantly lower adult height than AGA, whereas female SGA has no similar phenomenon. The growth rate of weight, height, and head circumference *Z* value of female children is greater than that of male children. The frontline growth can be promoted during adolescence, and the height can be normalized in early childhood. They maintain normal height in late childhood (Adolescence) and reach normal adult height.

### 2.4. Gestational Age Infant Data Set

The gestational age infant data include various indicators of the fetal parents' prepregnancy physical examination and postnatal follow-up surveys. The data are generated by researchers in various related fields across the country, including internal medicine, genetics, pediatrics, and family planning, and also science, public health, epidemiology, and the like. The coverage of the medical examination is extremely wide.

In the gestational age data obtained, the characteristics are mostly concentrated on the physical examination of the parents of the newborn fetus before pregnancy, including demographic information, including weight, height, blood type, cultural education, and ethnicity; the parents' usual living habits, such as whether they smoke or drink alcohol, whether to eat meat, and the like; the psychological status of the parents, such as whether there is financial pressure, whether there is work pressure; the parents' living environment factors, such as whether they are exposed to chemicals, radiation, and whether they have pets; the parent's reproductive system, such as male reproduction, and whether the organ is foreskin; the physical examination of the parents, such as blood pressure, urine routine, and the like.

At the same time, the original data of gestational age children cannot be directly put into the model for training. Directly using the original data for model training will lead to problems such as low efficiency of corresponding algorithm modeling and low accuracy. Therefore, the next task of this article is to preprocess the original data and normalize the data for model training.

Data cleaning: First, the original data are cleaned, and there are a large number of items that are of no use to the prediction of diseases of small-for-gestational-age infants. The detection items with too many missing values and the items with no value for disease prediction are deleted. Inspection features can be divided into two types: discrete features, such as blood type, family, and gender, using different codes to represent different attribute values in the features. Continuous features, such as blood pressure, creatinine, and other parental clinical physical examination items.

### 2.5. Model Building for Predicting Physical Growth

It is divided into two stages. The first stage is the unsupervised learning of the encoder, which is used for dimensionality reduction and abstraction of features. The second stage is to put the label of the sample into the model for supervised training, the purpose is to adjust the weight of the relevant parameters of the model.

The first stage is unsupervised learning. The input sample is an unlabeled sample, and the input layer and output layer of the model are the attribute values of the sample. At the same time, the hidden layer of the encoder is proved to be the best effect according to previous experiments. The main input data include date of birth, weight, maternal medical history, growth hormone, breast milk frequency, and protein content. In the improved encoder, it is necessary to add noise to the input layer because the proportion of noise will lead to the effect of feature dimensionality reduction and abstraction, and the accuracy of the supervised training classifier in the next stage.

The second stage is supervised learning. Fine tune the weights in the model, that is, add a classifier (Sigmoid layer) at the end of the unsupervised autoencoder, so that the unsupervised encoder has a classification function. The output of the model is compared with the label of the sample to perform supervised fine-tuning of the parameters.

## 3. Data Collection and Investigation

### 3.1. Sources of Information

Select children who are small for gestational age who are hospitalized in the neonatal intensive care unit from January 2020 to January 2021 and exclude children who are older than gestational age. The clinical hospitalization data were retrospectively analyzed and divided into two groups: early group and late group according to the relationship between gestational age and birth weight. The physical changes of these two groups of newborns were studied, and the incidence of SGA and AGA newborns in early and late premature infants was compared and analyzed.

### 3.2. Selection Criteria

The inclusion criteria were as follows:

1. The gestational age at birth is less than 37 weeks
2. The birth weight is below the 90th percentile of the average weight of infants of the same gestational age
3. The age at the time of admission is less than or equal to 24 hours

## 4. Result Analysis

### 4.1. General Situation

In this article, the male and female children accounted for 68% and 32%, respectively. Among them, 26%, 19%, 23%, and 11%, 8%, and 13% of early small for gestational age, midterm small for gestational age, and late small for gestational age, respectively, twin tires 32%, single tires 68%, as shown in Table 1.

As shown in Figure 2, we can know that there are more boys than girls and more single births than twins in small-for-gestational-age infants, and in terms of infant weight, low birth weight accounts for the largest proportion. Secondly, boys who are small-for-gestational-age in the early stage are the most born, followed by the late stage, while girls are born in the middle and late stages.

### 4.2. Comparison of the Incidence of Major Diseases in the Two Groups of Small for Gestational Age

The incidence in the early group was 52.1% for neonatal asphyxia, 22.5% for feeding intolerance, 14.8% for intracranial hemorrhage, 6.3% for scleredema, 24.7% for neonatal hyperbilirubinemia, 24.6% for hypoglycemia, 1.1% for apnea, and 3.2% for respiratory distress syndrome, as shown in Table 2:

As shown in Figure 3, the late group exhibited 41.3% of neonatal asphyxia, 11.9% of feeding intolerance, 5.6% of intracranial hemorrhage, 7.5% of scleredema, 33.8% of neonatal hyperbilirubinemia, 15.1% (38 cases) of hypoglycemia, 3.4% of apnea, and 1.3% of respiratory distress syndrome.

### 4.3. Postnatal Physical Development of Infants Younger than Gestational Age

When correcting gestational age, the incidence of growth deviations of underweight, growth retardation, microcephaly, overweight, and obesity were 21%, 12%, 3%, and 5%, respectively. The specific physical changes are shown in Table 3:

As shown in Figure 4, we can see that the highest incidence of growth retardation is 18% of corrected gestational age at 1 month, and the highest incidence of microcephaly, overweight, and obesity is 20% and 7% of corrected gestational age at 3 months. The incidence of low body weight (6%) after correction for 3 months was significantly reduced compared with correction for gestational age, and the difference was statistically significant (*P* < 0.05).

## 5. Conclusion

With the rapid advancement of computer technology, the standardization of data collection, and the rapid improvement of computing power, modern scientific research has brought new opportunities and support. Machine learning is one of the most important tools to bring new breakthroughs to the development of modern science. Machine learning is to discover potential mathematical laws from massive data and extract useful information to build related models. Based on computer data analysis technology, this article draws the following conclusions through experimental investigations: the survival rate of babies younger than gestational age is lower than that of normal babies; secondly, babies younger than gestational age have worse physique and are more likely to get sick. The growth process is more difficult, it is very likely that the intellectual development is not complete, the growth hormone is pitted, and the growth is not large. Children who are small for gestational age generally face the problem of insufficient nutrient intake in the early postnatal period. Due to insufficient fetal nutrition reserves, immature gastrointestinal function development, poor feeding tolerance, and other diseases after birth, it is still difficult to catch up with growth.

## Figures and Tables

**Figure 1:** Noise reduction autoencoder process.

**Figure 2:** Proportion of differences in gender and weight of SGA.

**Figure 3:** Comparison of the incidence of major diseases in the two groups of small-for-gestational age.

**Figure 4:** Postnatal physical development of SGA.

**Table 1:** Proportion of differences in gender and weight of SGA.

	SGA in the early stage (%)	SGA in the middle (%)	SGA in the late stage (%)
Male	26	19	23
Female	11	8	13
Twins	12	9	11
Single	21	25	22
Weight	29	62	9

**Table 2:** Comparison of the incidence of major diseases in the two groups of small for gestational age.

Principal disease	Early groups (%)	Late group (%)	*χ*2 value	*P* value
Asphyxia neonatorum	52.1	41.3	4.256	0.031
Feeding intolerance	22.5	11.9	4.765	0.021
Intracranial hemorrhage	14.8	5.6	5.437	0.021
Scleredema	6.3	7.5	0.198	0.654
Hyperbilirubinemia	24.7	33.8	2.138	0.129
Glucopenia	24.6	15.1	4.389	0.032
Apnea	1.1	3.4	0.743	0.356
RDS	3.2	1.3	0.324	0.457

**Table 3:** Postnatal physical development of SGA.

Correct the month age	Low weight case (%)	Growth retardation example (%)	Microcephaly cases (%)	Overweight (%)
0	21	12	3	5
1	6	18	10	7
3	6	10	20	7
6	11	4	2	1

## Data Availability

The data underlying the results presented in the study are available within the manuscript.
